This article has been retracted.

# Application of Intelligent Image Matching and Visual Communication in Brand Design

**DOI:** 10.1155/2022/5964851

**Published:** 2022-08-05

**Authors:** Ming Liu, Wenyan Zhong

**Affiliations:** ^1^School of Communication and Design, Longyan University, Longyan 364000, China; ^2^Department of Design, Hainan Vocational University of Science and Technology, Haikou 571126, China

## Abstract

In this paper, from the perspective of improving the visual communication of brand design, image texture intelligent matching processing is needed, proposing a brand design texture intelligent matching method based on visual communication, constructing a brand design texture intelligent information acquisition model under visual communication, using automatic image imaging technology for texture imaging and feature segmentation of brand design, and extracting typical brand design and ethnic design language of texture histogram, texture segmentation, and automatic matching under visual communication according to histogram distribution, brand design texture information enhancement and optimization detection by regularized feature fusion method, extraction of edge contour feature points of brand design, and texture matching with the extracted edge contour feature points of decorative patterns as input statistics. The adaptive performance of texture matching for a brand design using this method is better, and the texture discrimination ability is stronger, which improves the application research of better reflecting brand design in modern visual communication design and promotes the innovative combination of traditional cultural elements and modern design.

## 1. Introduction

The concept of visual packaging design is to give the audience visual and psychological cognition from words, graphics, and colors [1]. It establishes the logo, color, and labeling and is used for identification shorthand. For consumers, brand perception is the most beneficial tool to judge and distinguish similar products. The brand is used to reduce the time to choose [2].

A dazzling visual packaging war was staged between TV stations and channels. In the midst of the audiovisual inundation but can not help but disappoint some people. The form does not focus on positioning but only seeks to obtain gorgeous visual effects [3]. In the competition of brand media, not only the formal beauty should be pursued but also the connotation of the theme and the brand effect should be added [4]. The impact of digital packaging on the brand of television media and the important role of brand image [5]. Through the analysis and systematic elaboration of the packaging process. Misconceptions, drawbacks, and successful columns are taken as the focus of the analysis. To explore the role of media packaging and excellent columns for brand building [6]. Learn from successful packaging and make the production team brand conscious as well through brand awareness implantation [7]. It is important to consider not only positioning, style, and innovation, but also brand awareness in production [8].

Speaking of packaging seems to know what he means, and it has a lot in common with the usual packaging of products. Packaging is also borrowed for the packaging of products. And, the definition of TV packaging is the specification and strengthening of the audiovisual elements of the channel, column, and TV station image as a whole [9]. Packaging design prerequisites are to solve the audience for their channel and the initial recognition of the column and program identification superior poor choice. Such as a channel to broadcast a new TV series in prime time, before the broadcast to be after the packaging design to edit out the exciting images of the TV series, story conflict, in the postvisual design as a TV series promotional video [10]. Publicity to the audience, this is not the era of good wine is not afraid of the alley, is the need for active marketing and self-promotion of the times [11]. For the status of their own brand, the establishment of personality characteristics is the audience to establish their own channel media must mean of recognition [12].

Packaging is an important part of media brand building. In an era of excessive selectivity, you are successful if you catch the audience's eye, while hasty conversion is your undoing. For viewers to choose you, an initial understanding of you is essential. In addition to the full publicity on the TV screen [13]. This is not enough, in the development of the network today, the popularity of smart phones, tablets, the network, and cell phone platform publicity when it is the way to go. TV media need to actively promote the network if they want to break through [14]. By bringing PPS videos close to other smartphones and tablets so that they are no longer limited by space, the visual packaging design of the media is the most direct means of publicity for each platform [15].

This is not conducive to the interests of the channel itself, so it is generally more stable, and if there are changes, they are modified and improved in the initial design [16]. We try to keep the original features and optimize only in terms of beautification. For example, the image logo of Phoenix TV is two phoenixes flying together. This logo leaves a deep impression, and whenever you see this logo you will clearly identify this Phoenix TV. Excellent LOGO image will make the audience remember deeply and penetrate into the audience's mind. A fixed memory is formed. When choosing a channel, based on the label viewers will quickly choose what frequency to see [17]. What programs are available on the channel and which ones do they like. Through tags, viewers can establish a connection. The label is in the upper left corner of the screen, which has become an inherent pattern in the media, as a necessary element that is inherent on the TV screen in addition to being fixed on the screen. There is a digital visual design of dynamic video often referred to as logo rendering that scrolls between programs in the channel [18]. When creating the logo image, attention should be paid to simplicity and clarity, outstanding features, reflecting modernity and design, incorporating regional culture, and enhancing viewability and locality [19]. In the channel, the interpretation of LOGO can enhance the sense of coherence between programs, make the rhythm and paragraphs more compact, and fill the gap between programs and advertisements. In media packaging, dynamic LOGO interpretation and image logo design are the cornerstones of tonality and make the features more prominent [20].

## 2. Image Acquisition and Preprocessing of Brand Texture Patterns

### 2.1. Image Acquisition of Brand Texture Pattern

In order to realize the intelligent matching of brand design texture based on visual communication, firstly, the 3D image reconstruction method is used for visual information acquisition of brand texture pattern, and the multimedia digital information reconstruction method is used for intelligent matching of brand design texture, visual feature sampling, and the intelligent matching of brand design texture in the texture distribution area of the image; the image feature reconstruction space technique is used to read the 3D of brand design texture data feature volume, and form the raw file of brand design texture, the brand design texture PBO (OpengGl pixel cache object) is built according to the spatial feature sampling technique, and the image is stored in device memory, the brand design texture information is read, and the brand design texture matching is performed according to the brand design data information in device memory. According to the above-given design idea, it is assumed that the pixel set distribution of brand texture pattern is *n*, and the amount of label category information features of the output brand texture pattern is *P*(1)=[1 − *L*^−1^]*m* − 1. According to the size and texture complexity of the brand design, the brand texture point pair matching is performed to get the brand texture pattern texture distribution.

(1) $$\begin{array}{c} E_{m}^{ij}=\sum_{k=0}^{255}e_{mk}^{ij}, \end{array}$$

where *E*_*m*_^*ij*^ is the color information of column *j* of row *i* in the *m* th image of the 3D branded texture pattern data sampling sequence.

(2) $$\begin{array}{c} e_{mk}^{ij}=\left\{\begin{array}{cc} -p_{k}\log\left(p_{k}\right) & p_{k}\neq 0\\ 0 & p_{k}=0 \end{array}\right\}. \end{array}$$

Here, *e*_*mk*_^*ij*^ for the 2 × 2 brand design edge information.

Combining the pixel frame distribution for texture alignment, the brand texture pattern information is fused using *k* th order moment feature statistics for the pixel points on each scale *σ*_*I*_^(*n*)^(1,2,…, *n*), and one sampling point is taken in each subinterval to obtain the grayscale histogram of the brand texture pattern.

(3) $$\begin{array}{c} P_{k}=\frac{n_{k}}{\sum_{i=0}^{255}n}. \end{array}$$

For *N* brand design labels, the information fusion expression for the color, texture, shape, and other features of the brand texture pattern is

(4) $$\begin{array}{c} c\left(x,y\right)=\left[\begin{array}{cc} \Delta x & \Delta y \end{array}\right]\left[\begin{array}{cc} \sum_{W}I_{x}^{2} & \sum_{W}I_{x}I_{y}\\ \sum_{W}I_{x}I_{y} & \sum_{W}I_{y}^{2} \end{array}\right]\left[\begin{array}{c} \begin{array}{c} \Delta x\\ \Delta y \end{array} \end{array}\right]. \end{array}$$

The intelligent information acquisition model of brand design texture under visual communication is constructed, and the automatic image imaging technology is used for texture imaging and feature segmentation of brand design, and the average energy of the window is examined, and the neighborhood frame intensity at the spatial scale of brand design texture at (*x*, *y*, *σ*) is

(5) $$\begin{array}{c} H=\left[\begin{array}{c} L_{xx}\left(x,\sigma \right)L_{xy}\left(x,\sigma \right)\\ L_{xy}\left(x,\sigma \right)L_{yy}\left(x,\sigma \right) \end{array}\right], \end{array}$$

where *L*_*xx*_(*x*, *σ*) is the brand design texture convolution, *L*_*xy*_ and *L*_*yy*_ have similar meanings. According to the fusion result of the edge pixel set of brand design, the multidimensional feature space reconstruction method is implemented for brand texture pattern information collection, and the edge energy value of the regional distribution pixel points *p*(*i*, *j*) of brand design is obtained, which is used as the data input basis for intelligent matching and feature extraction of brand design texture.

### 2.2. Brand Design Feature Segmentation

The automatic image imaging technology is used for texture imaging and feature segmentation of the brand design, and the texture histogram of the brand design is extracted. According to the known pixel points *x* of the brand texture pattern, the maximum intensity of the texture distribution of the brand texture pattern is obtained to satisfy *I*(*x*)=1, and the regional template matching the value of the brand image is determined as follows:

(6) $$\begin{array}{c} I_{\text{total}}=\frac{L_{\text{total}}}{\rho_{SRm}\left|S_{SR}\right|}\\ =\frac{\sum_{i=1}^{M}\sum_{m=1}^{\left|S_{SR}\right|}\left(\lambda_{i}p_{im}T_{SRm}/\rho_{SRm}\right)}{\left|S_{SR}\right|}. \end{array}$$

The adaptive chunking feature matching method is used to determine the priority coefficients of the branded texture pattern output, and the dyadic geometric relationship of the output branded texture pattern is described by the following equation:

(7) $$\begin{array}{c} P=\sum_{i=1}^{M}\left(\lambda_{i}•\frac{\sum_{m=1}^{\left|S_{SR}\right|}p_{im}T_{SRm}}{\sum_{m=1}^{\left|S_{SR}\right|}\lambda_{SRm}}\right). \end{array}$$

The template alignment of the branded texture pattern is performed using the texture intelligent matching method, and the template alignment function is constructed as follows:

(8) $$\begin{array}{c} \text{STFT}\left(t,f\right)=\int_{-\infty }^{\infty }x\left(\tau \right)h^{*}\left(\tau -t\right)e^{-j2\pi f\tau }\text{d}\tau . \end{array}$$

Using the pixel difference between the two branded texture patterns *K*_*m*_ and the spatial distribution pixel level *s*, the branded texture matching window is

(9) $$\begin{array}{c} \text{SPEC}\left(t,f\right)={\left|\text{STFT}\left(t,f\right)\right|}^{2}. \end{array}$$

Using the adaptive chunking technique, a brand design texture template matching window of 2^*l*^ times the length and width is created, and the brand design texture distribution function is described as follows:

(10) $$\begin{array}{c} U\left(x\right)=1-{\tilde{t}}^{\prime }\left(x\right)\\ =\omega \tilde{U}\left(x\right)\\ =\omega \min_{c\in \left\{r,g,b\right\}}\left(\min_{y\in \Omega \left(x\right)}\left(\frac{I^{c}\left(y\right)}{A}\right)\right). \end{array}$$

The brand design texture segmentation is performed by means of a two-dimensional function expression, and the schematic diagram of the implementation process is shown in Figure 1.

## 3. Brand Design Texture Intelligent Matching Optimization

### 3.1. Texture Histogram Extraction of Brand Design

Based on the above-mentioned construction of the intelligent information collection model of brand design texture under visual communication, the intelligent matching of brand design texture is carried out, and a method of intelligent matching of brand design texture based on visual communication is proposed. With the feature points of edge texture distribution as the center, the fuzzy feature distribution function of the brand texture pattern is calculated in the irregular texture distribution triangle region *W*_*mE*_^*ij*^. The initial pixel set of the brand design is described as follows:

(11) $$\begin{array}{c} L\left(a,b_{m}\right)=\sum_{V_{m}\in P_{\text{res }}^{n}\in }\in \sum_{\text{Prtue }}\frac{\left|V_{m}\cap V_{n}\right|}{\left|V\right|}\log\left(\frac{\left|V\right|\left|V_{m}\cap V_{n}\right|}{\left|V_{m}\right|\left|V_{n}\right|}\right). \end{array}$$

The scale function of the distribution of feature points of the brand design is obtained and expressed as follows:

(12) $$\begin{array}{c} W_{mE}^{ij}=\frac{E_{m}^{ij}}{\sum_{m=1}^{N}E_{m}^{ij}}. \end{array}$$

Within the grayscale neighborhood of the brand design, the spatial distribution of texture-matched clusters with center lengths of

(13) $$\begin{array}{c} d_{mn}^{ij}\left(x,y\right)=\left\{\begin{array}{cc} \frac{\sum_{k=-s}^{+s}\left|\theta_{m}^{ij}\left(x+k,y+k\right)-\theta_{n}^{ij}\left(x+k,y+k\right)\right|}{{\left(2s+1\right)}^{2}}, & m\neq n,\\ 0, & m=n, \end{array}\right. \end{array}$$

where *m*, *n* are the image projection numbers of the brand texture pattern in 3D; *i*, *j* are the feature matching points of the brand texture pattern; *θ* is the regional rotation angle of the brand texture pattern.

The Taubin smoothing operator is used to reconstruct the brand texture pattern in 3D, and the main directional feature components of the edge contour of the brand texture pattern are noted as follows:

(14) $$\begin{array}{c} D_{mn}^{ij}\left(x,y\right)=\left\{\begin{array}{cc} 1, & d_{mn}^{ij}\left(x,y\right)\geq \mathrm{median}\left(d_{mn}^{ij}\left(x,y\right)\right),\\ 0, & \text{others,} \end{array}\right. \end{array}$$

where median() is the median operation expression, and the texture matching value *W*_*mD*_^*ij*^ is obtained according to the sparsity of the boundary pixel points of the brand design.

(15) $$\begin{array}{c} W_{mD}^{ij}=\left\{\begin{array}{cc} 1, & n_{md}^{ij}<\alpha ,\\ 0, & \text{othes}, \end{array}\right. \end{array}$$

where *n*_*md*_^*ij*^ is the set of edge pixels of the brand design; *α* is the ratio of the number of all pixels, set at 5%.

### 3.2. Visual Communication of Brand Design

Constructing the texture activity contour component of the brand design in the 4 × 4 subgrid region, setting *h* as the edge pixel set of the brand design, using the adaptive chunking feature matching method for window template matching, and using *w*_*i*_ as the weighting vector within the *N* × *N* window, the center pixel set and edge pixel set of the brand design is expressed as follows:

(16) $$\begin{array}{c} I_{if}\left(x,y\right)=I^{*}G\left(x,y,\sigma_{i}\right),\\ I_{iv}\left(x,y\right)=I^{*}\text{stdfilt}\left(x,y,w_{i}\right),\\ S_{gif}\left(x,y\right)=-\log\left(P_{if}\left(x,y\right)\right), \end{array}$$

where *G*(*x*, *y*, *σ*_*i*_) is the multichromatic set of the brand design, and the texture matching hierarchy function of the brand design is calculated at each scale *σ*_*I*_^(*n*)^(1,2,…, *n*) of the brand design.

(17) $$\begin{array}{c} L\left(a,b_{m}\right)=\log\left(\frac{\left|V\right|\left|V_{m}\cap V_{n}\right|}{\left|V_{m}\right|\left|V_{n}\right|}\right). \end{array}$$

According to the feature segmentation of the edge contour feature points of the image, the fusion feature distribution of the decorative pattern is obtained as follows:

(18) $$\begin{array}{c} f_{R}\left(z\right)=\left(\begin{array}{c} f_{x}\left(z\right)\\ f_{y}\left(z\right) \end{array}\right)=\left(\begin{array}{c} h_{x}*f\left(z\right)\\ h_{y}*f\left(z\right) \end{array}\right), \end{array}$$

where *f*(*z*) is the texture feature component of the brand design and *∗* is the convolution operation.

The amount of edge information features of the brand design is calculated, and the optimized brand design feature extraction output is obtained as follows:

(19) $$\begin{array}{c} E\;\mathrm{int}\left(vi\right)=\frac{1}{2}\left(\partial i\;{\left|d-\left|vi-vi-1\right|\right|}^{2}+\beta i{\left|vi-1+2vi+vi+1\right|}^{2}\right), \end{array}$$

where

(20) $$\begin{array}{c} d=\frac{1}{n}\sum_{i=0}^{n-1}\left|vi-vi-1\right|. \end{array}$$

Let *I*_*x*_ be the chunked feature matching set of the brand design, where *x*=*P*, *N*, The activity profile of the brand design is

(21) $$\begin{array}{c} S_{c}={\left[S_{0},\ldots ,S_{Q-1}\right]}_{\text{binary}}={\left[\sum_{i}^{Q-1}S_{i}\times 2^{i}\right]}_{\text{Dec}},\\ S_{i}=\sum_{j}^{W\times W}I_{x}^{j}, \end{array}$$

where *Q* is the edge scale of the brand design; *W* is the amount of weak edge features.

The regularized feature fusion method is used for brand design texture information enhancement and optimal detection, and the output texture intelligent matching map is obtained as follows:

(22) $$\begin{array}{c} w\left(i,j\right)=\frac{1}{Z\left(i\right)}\exp\left(-\frac{d\left(i,j\right)}{h^{2}}\right), \end{array}$$

where *Z*(*i*)=∑_*j*∈Ω_exp(−(*d*(*i*, *j*)/*h*^2^)) is the symbolic distance function of brand design feature extraction, and let *H*_*x*_, *H*_*y*_ be the wavelet feature solution of multiresolution brand design, respectively, to obtain the chromatographic distribution matrix of the image as follows:

(23) $$\begin{array}{c} C=O^{T}O\left[\begin{array}{c} \sum H_{x}\left(t\right)H_{x}\left(t\right)\sum H_{x}\left(t\right)H_{y}\left(t\right)\\ \sum H_{y}\left(t\right)H_{x}\left(t\right)\sum H_{y}\left(t\right)H_{y}\left(t\right) \end{array}\right]. \end{array}$$

Using the extracted edge contour feature points of the decorative pattern as input statistics for texture matching, the texture matching output is obtained as follows:

(24) $$\begin{array}{c} O=USV^{T}, \end{array}$$

where *U* is the matrix of pixel training sample set of brand design in *N* × *N* dimensions, and in summary analysis, the intelligent matching of brand design texture based on visual communication is achieved [21, 22].

## 4. Brand Design Effect

There are many different forms of design in digital visual design packaging. Among the many variations, there are also fixed patterns. For modular packaging, the first and foremost is the channel promo. It has many styles, such as brand presenter image propaganda and regional cultural elements propaganda. There are also abstract picture combinations, national elements of traditional painting art, and postmodern three-dimensional post-technology synthesis style show. CCTV's “power of brand” is of great significance to the channel's promotional video. Delicate production, from ancient to the contemporary use of elements: interspersed, ink, ink splash, the use of techniques. It has to be said that it is deeply appealing. The creative form is based on the style of Chinese ink and wash, with the regional landmarks of Greater China. To witness the rise of China and the road to the realization of the Chinese dream. This not only represents the brand of the channel media. It also reflects the disgusted Chinese culture and the rise of the nation. It is a window to the world to declare our dream and the belief to achieve it. It further establishes the cultural communication concept of CCTV and its own brand image. As shown in Figure 2.

Various different channels and different columns in their promotional video production methods also have a lot of different strategies. Such as CCTV's windmill column have mostly children as the audience. Then, it is the pursuit of fantasy, science fiction, and childlike. His style of production, can not be limited to the host of the promo class. More to join the digital technology now three-dimensional animation effects, to produce a fantastic and bizarre fairy tale world to make it more attractive. Fully demonstrate the whimsical mode of thinking of children. In combination with specific channel call signs, etc., such as the CCTV13 news channel, its promos, and headlines are mostly in the image of reporters and hosts for real-time interview documentary. The picture switches quickly, which makes the content more realistic, comprehensive, and global [23, 24].

In short, each program has its own positioning and presentation. It is the best to seize its own characteristics and find the suitable form of expression as shown in Figure 3.

A place of water and soil nurtures a place of people. This is also true for television media. However, this is also true for digital visual design. The characteristics of the region's packaging can always resonate with the region. For example, in the packaging design of Jinan TV, the application elements always revolve around the characteristics of the spring city. With water and springs, plus the city flower of Jinan. It not only reflects the regional characteristics. Also, for the city to make favorable publicity. For other provinces and cities, according to the different geographical location, cultural background, and ethnic folklore to package themselves to establish a unique style. In the design of highlighting the personality and regional characteristics, folk culture is one of the inevitable choices of the principle of characteristics as shown in Figure 4.

## 5. Experimental Results and Analysis

In order to verify the overall effectiveness of the self-matching method of significant image feature weights based on visual communication. The hardware environment during the test was an AMDA6-36702.70 GHz CPU, and the computer's memory was 2G The operating system is MatlabR2010b [25].

The time used to match the image feature weights by the three different methods was compared, and the test results of the three different methods are shown in Figure 5.

Analysis of Figure 5 shows that the matching time used in multiple iterations is less than 3 s when the significant image feature weight self-matching method based on visual communication is used to match the image feature weights; analysis of the matching time used in multiple iterations fluctuates around 5 s when the image feature weight self-matching method based on median filtering and the image feature weight self-matching method based on percolation filter are used to match the image feature weights. The matching time used in multiple iterations fluctuates around 5 s when matching. The test results show that the self-matching method of significant image feature weights based on visual communication takes less time to match the image feature weights because the self-matching method of significant image feature weights based on visual communication uses the linear combination of filter functions to represent the response of the filter, which reduces the number of convolution operations, decreases the amount of operations, and shortens the time used for self-matching the image feature weights, verifying that the self-matching method of significant image feature weights based on visual communication. It is verified that the matching efficiency of the significant image feature weight self-matching method based on visual communication is high.

The image feature weight self-matching method based on the percolation filter are tested, and the matching accuracy of the three different methods is shown in Figure 6.

According to the analysis of Figure 6, the matching accuracy is around 90% in multiple iterations. According to the analysis of Figure 6, the matching accuracy of the self-matching method based on the median filter fluctuates around 80% in multiple iterations. According to the analysis of Figure 6, the matching accuracy of the self-matching method based on an osmotic filter fluctuates around 70% in multiple iterations.

According to the above-given analysis, the matching accuracy of the self-matching method based on visual communication is higher than that of the self-matching method based on median filter and the self-matching method based on an osmotic filter. Because the self-matching method of significant image feature weight based on visual communication constructs a controllable filter to extract image features, reduces repeated convolution operations, solves the problem of poor subjective visual effect caused by human eye sensitivity, realizes the matching of image feature weight through the ratio method, and improves the matching accuracy of the method.

## 6. Conclusion

The significance of digital packaging lies in the promotion of the brand. In the process of packaging, publicity, and communication, make the potential output of media concept culture. The audience is unconsciously affected. Digital packaging only beautifies and conveys. Based on the application of the image matching method and visual communication in brand design, this paper is an effective platform to establish a brand and expand the business. At the same time, promote their own value and enhance the brand image of the media.

## Figures and Tables

**Figure 1:** Schematic diagram of the implementation process of brand design texture segmentation.

**Figure 2:** Brand image.

**Figure 3:** Brand image.

**Figure 4:** Cultural image.

**Figure 5:** Matching time of three different methods.

**Figure 6:** Matching accuracy of three different methods.

## Data Availability

The experimental data used to support the findings of this study are available from the corresponding author upon request.
